# Tumor Necrosis Factor-Alpha Disrupts Cx43-Mediated Corneal Endothelial Gap Junction Intercellular Communication

**DOI:** 10.1155/2022/4824699

**Published:** 2022-09-19

**Authors:** Jufeng Meng, Ke Xu, Yinyin Qin, Ya Liu, Lin Xu, Shigang Qiao, Jianzhong An, Jianjun Liu, Zhenhao Zhang

**Affiliations:** ^1^School of Life Science and Technology, ShanghaiTech University, Shanghai 201210, China; ^2^Key Laboratory of Tropical Translational Medicine of Ministry of Education, NHC Key Laboratory of Control of Tropical Diseases, School of Tropical Medicine, Hainan Medical University, Haikou 571199, China; ^3^Institute of Clinical Medicine Research, Suzhou Science & Technology Town Hospital, Suzhou 215153, China; ^4^Department of Ophthalmology, Suzhou Science & Technology Town Hospital, Suzhou 215153, China

## Abstract

Connexin43 (Cx43)-mediated gap junctions are vital in maintaining corneal endothelium homeostasis. Tumor necrosis factor-alpha (TNF-*α*) is among the most important inflammatory factors which cause corneal endothelial dysfunction in various eye diseases. However, the effect of TNF-*α* on Cx43-mediated gap junctions of the corneal endothelium remains undefined. In the current research, we determined the effect of TNF-*α* on gap junction intercellular communication (GJIC) in rabbit corneal endothelium. To evaluate alterations of GJIC, if any, we treated ex vivo cultured rabbit corneal endothelium with different concentrations of TNF-*α* (2-20 ng/ml). The localization of Cx43 was analyzed by immunostaining, while RT-qPCR and western blot were used to profile the expression of Cx43 and zonula occludens-1 (ZO-1). The association between ZO-1 and Cx43 was evaluated using immunoprecipitation and double staining. GJIC activity was determined by the scrap loading and dye transfer assay (SLDT). Our data demonstrated that a high concentration of TNF-*α* (10 ng/ml and 20 ng/ml) disrupts the Cx43 mediated gap junction distribution in rabbit corneal endothelium and suppresses the expression of Cx43 protein. Furthermore, rabbit corneal endothelial GJIC was inhibited due to the decreased association between the ZO-1 and Cx43 proteins. Current results demonstrate that TNF-*α* inhibits corneal endothelial GJIC via decreasing the association between ZO-1 and Cx43, disrupting the distribution of Cx43, and downregulating the expression of Cx43 protein. This study offers a new theoretical foundation for diagnosing and treating corneal endothelial cell decompensation induced by elevated TNF-*α* in various eye diseases.

## 1. Introduction

With the increase in age, the density of human corneal endothelial cells reduces by 0.6% annually [1]. Following insults such as intraocular surgical trauma, topical application of drugs, and corneal transplantation, the cell cycle is arrested at the G1 phase and fails to proliferate in vivo [2]. In endothelial cells of patients with decompensation, corneal endothelial transplantation is the best treatment option. However, the lack of donors and low survival rate after corneal endothelial transplantation severely limit the wide clinical development of corneal transplantation. To circumvent this challenge, there is a critical need to study the homeostasis of the corneal endothelium. Under normal physiological circumstances, gap junction channels made of 2 connexons that dock between corneal endothelial cells can allow small molecular nutrients, signal compounds, like inositol trisphosphate (IP3), nucleotides, and Ca^2+^, as well as metabolites, to pass through and perform intercellular communication, thus playing a key role in maintaining the internal environment and metabolism of the corneal endothelial cells [3, 4]. Connexon is composed of six connexin subunits [5], and 21 different types of connexins have been identified to date. Out of the various types of connexins, connexin43 (Cx43) has been the most studied and widely distributed gap junction protein. The Cx43 protein is the most common connexin subtype expressed in bovine [4], human [6], rabbit [7], and rat corneal endothelial cells [8]. Our previously published results also confirm that Cx43 plays an important role in maintaining the homeostasis of GJIC in rabbit corneal endothelial cells [9]. Gap junctions can influence cell death and survival responses to oxidative and metabolic stress [10]. However, dysfunction of Cx43-mediated gap junction intercellular communication (GJIC) induces many diseases, including cardiovascular diseases [11], neuropathy [12], cancer [13], and ocular diseases [14].

Connexin family members have a half-life of 2-5 h and undergo gap junction plaque organization to final degradation in this process [3]. However, the specific mechanisms that regulate the assembly and degradation of gap junctions remain poorly understood. It is reported that Cx43 binds to PDZ domain of ZO-1 through the C-terminal domain to maintain the dynamic balance of gap junction [15]. The ZO-1 protein not only helps organize gap junction plaques but also participates actively in Cx43 trafficking and internalization, and thereby exerts biological effects [16]. Meanwhile, phosphorylation of Cx43 regulates gap junction plaques organization and GJIC activity [17].

Inflammatory factors in aqueous humor induced by endophthalmitis, uveitis, ocular trauma, and other ocular surgeries lead to corneal endothelial dysfunction, thus affecting the metabolism of endothelial cells and maintenance of the internal homeostasis [18, 19]. TNF-*α* is one of the most important inflammatory factors which causes corneal endothelial impairment and is crucial in immune regulation [20]. Hao et al. and Kimura et al. showed that TNF-*α* inhibits Cx43-mediated GJIC activity by activating JNK signaling pathway in cultured human corneal fibroblasts, suggesting that the JNK pathway can regulate the functions of the gap junction [21, 22]. The study also showed that TNF-*α* can induce Cx43 degradation by the ubiquitin-proteasome pathway and can inhibit the GJIC activity of corneal fibroblasts [23]. Our previous study have found that TNF-*α* disrupts the corneal endothelial barrier function maintained by tight junction protein ZO-1 by promoting myosin light chain (MLC) phosphorylation [24]. Another study demonstrated that preservative benzalkonium chloride (BAK) inhibits GJIC by phosphorylating Cx43 and downregulating Cx43 expression [9]. Although several studies on TNF-*α* and corneal gap junction have been carried out, the effect of TNF-*α* on Cx43-mediated gap junctions of the corneal endothelium remains unclear. In this study, our data showed that in ex vivo cultured rabbit corneal endothelial tissue and primary cultured rabbit corneal endothelial cells, treatment with high concentration of TNF-*α* (10, 20 ng/ml), could disrupt GJIC via attenuating the association between ZO-1 and Cx43 proteins as well as disrupting the distribution of Cx43 and decreasing the expression of Cx43.

In summary, this study demonstrated how rabbit corneal endothelial cells respond to TNF-*α* stimuli and showed changes in the GJIC. The current results highlight a novel molecular mechanism underlying the damage to corneal endothelial functions caused by increased TNF-*α* in various eye diseases. Thus, targeting the gap junctions could be a novel strategy to protect the corneal endothelium.

## 2. Materials and Methods

### 2.1. Animals

The Shanghai SLAC Laboratory Animal Co., Ltd. (Shanghai, China) provided us with male New Zealand white rabbits weighing between 1.5 and 2 kg each (Shanghai, China). The animals were fed in a standard environment at 20 ± 1°C, and the lighting was simulated day and night. All experiments on animals have been performed in accordance with the guidelines of ARVO for Ophthalmic and Vision Research and were authorized by the Laboratory Animal Council of the Suzhou Science and Technology Town Hospital.

### 2.2. Reagents and Antibodies

DMSO and Triton X-100 were purchased from Abcone (Shanghai, China). Pentobarbital sodium, TNF-*α*, and Lucifer yellow dye were obtained from Sigma-Aldrich (St. Louis, MO). Primary ZO-1 antibody (mouse anti-rabbit), donkey anti-mouse IgG Alexa Fluor 488, and donkey anti-goat IgG Alexa Fluor 555 were purchased from Thermo Fisher Scientific (Carlsbad, CA). Santa Cruz (Santa Cruz, CA) provided goat-anti-rabbit Cx43 antibodies; HRP-conjugated donkey anti-goat IgG was from Bio-Rad (Hercules, CA). HUABIO (Hangzhou, China) supplied mouse anti-rabbit *β*-actin antibody, whereas Bio-Rad supplied HRP-conjugated goat anti-mouse IgG (Hercules, CA). Magnetic protein G beads and protein A/G beads were from Millipore (Billerica, MA) and Bimake (Houston, TA) ,repectively. PVDF membrane and 0.25% Trypsin-EDTAwere obtained from Thermo (Carlsbad, CA); ECL kit was provided by Shanghai Epizyme Biomedical Technology Co., Ltd (Shanghai, China); DAPI-mounting media were provided by Vector Laboratories (Burlingame, CA); BSA powders and collagenase I were acquired from Sangon Biotech (Shanghai, China) while DMEM, DMEM/F12, FBS, and Penicillin-Streptomycin (PS) were obtained from Thermo (Carlsbad, CA).

### 2.3. Ex Vivo Culture of Rabbit Corneal Endothelial Tissue Layers

After the rabbits were euthanized, the corneal epithelial cells were carefully scraped under a stereomicroscope (Olympus, Japan), and then venus scissors were employed to remove the remaining corneal tissue along the limbus. Isolated rabbit corneal endothelial tissue layers were grown in DMEM supplemented with 10% FBS and 1% PS as our previously reported study. The corneal endothelial tissue layers were then exposed to different concentrations of TNF-*α* (2-20 ng/ml) in a humid environment that included 5% CO_2_ at 37°C for 24 h. On the other hand, ex vivo cultured rabbit corneal endothelial tissue layers without TNF-*α* treatment were used as normal controls.

### 2.4. Immunostaining

After TNF-*α* (0-20 ng/ml) treatment at 4°C, rabbit corneal endothelial tissue layers were promptly fixed with 4% paraformaldehyde for 15 minutes. Following three washes cycles using TD buffer solution (PBS containing Triton 1% and DMSO 1%), a nonspecific interaction was inhibited by incubating tissues with BSA 2% at RT for 60 min. The rabbit corneal endothelial tissue layers were then incubated with goat anti-rabbit Cx43 polyclonal antibody (Santa Cruz) or polyclonal ZO-1 antibody (Thermo), then was diluted in BSA 1% and kept at 4°C overnight. Thereafter, the tissues were subject for 3 cycles of washing using PBS, and then it treated at RT for 60 minutes using different secondary antibodies (donkey anti-goat IgG Alexa Fluor 594 conjugated, goat anti-rabbit Alexa Fluor 488 conjugated, both diluted 1 : 300 in 1 percent BSA). Following a 3 washing cycle utilizing PBS, 4 incisions were performed in the cornea, and DAPI staining was performed on the endothelial tissues of the cornea. The slices were viewed under a confocal laser scanning microscope (CLSM, Zeiss 880) and then photographs were processed and investigated utilizing Zeiss Blue software.

### 2.5. Western Blot

The isolated rabbit corneal endothelial tissue layers were washed 3 times in a phosphate buffer saline before being lysed in RIPA buffer solution containing protease inhibitor 1% (Thermo). The concentration of the proteins was measured using a BCA protein kit (Beyotime Biotechnology, Shanghai, China) via centrifuging at 14000 g for a half-hour at 4°C. After SDS-PAGE separation, the proteins were transported to membranes of PVDF. At room temperature, the membranes were blocked with TBST that was supplemented with 2% BSA. After that, the membranes were incubated with primary anti-ZO-1, Cx43, or anti-actin antibodies at 4°C in TBST that contains 1% BSA. Thereafter, membranes were incubated with the secondary antibodies at room temperature for 1.5 hours. After washing 3 times with TBST, the blots were exposed to ECL reagents for visualization of immunocomplexes. An image analysis software package was used to analyze the band intensities with a gel imaging system (Bio-Rad, CA).

### 2.6. RT-qPCR Analysis

The rabbit corneal endothelial layers were isolated under a surgical microscope as previously described. Total RNA of the corneal endothelium was extracted with EasyPure RNA kit and then adjusted to the same concentration. Subsequently, the Reverse Transcriptase kit (Vazyme biotech, China) was used to synthesize cDNA from the extracted RNA, which was then amplified using an SYBR qPCR Mix kit (Vazyme biotech, China) in a QuantStudio 5 PCR instrument (Thermo, USA) using specific primers for Cx43, ZO-1, and GAPDH. Following are the PCR primer sequences: ZO-1 (forward, 5′-GTCTGCCATTACACGGTCCT-3′ reverse, 5′-GGTCTCTGCTGGCTTGTTTC-3′), Cx43 (forward, 5′-GCAAGCTCCTGGACAAAGTC-3′, reverse, 5′-CGTTGACACCATCAGTTTGG-3′), and GAPDH (forward, 5′-ACCACAGTCCACGCCATCAC-3′, reverse, 5′-TCCACCACCCTGTTGCTGTA-3′). The mRNA expression profiles were assessed utilizing the ΔΔCT technique, then standardized to rabbit GAPDH.

### 2.7. Immunoprecipitation

Fresh isolated rabbit corneal endothelium were homogenized in immunoprecipitation buffer and lysed on ice for 2 h. Protein concentration was determined after centrifugation at 16000 g for 35 min at 4°C for cell lysates. Magnetic protein G beadswere used to remove nonspecific binding for 1 h at RT. After removing the magnetic beads, the supernatant was incubated overnight with primary Cx43 antibody and protein A/G beads. Thereafter, the beads were collected by centrifugation at 18000 g for 18 min at 4°C and washed 4 times with immunoprecipitation buffer. The proteins bound to the magnetic beads were denatured by heating at 100°C, followed by immediate WB analysis as described above.

### 2.8. Primary Rabbit Corneal Endothelial Cells Culture and SLDT Assay

GJIC activity can be analyzed using SLDT assay by measuring the distance, the dye permeates through gap junction, or calculating how many dye-containing cells there are. In order to effectively evaluate GJIC activity, primary cultured corneal endothelial cells were used in this study to analyze the effect of TNF-*α* on GJIC. Firstly, isolated rabbit corneal endothelial layers were digested overnight at 37°C by 10 mg/ml collagenase I, followed by treatment with 0.25% trypsin-EDTA for 5 minutes to break up into single cells. When primary rabbit corneal endothelial cells cultured in DMEM/F12 supplemented with 10% FBS and 1% PS reached to 70% confluence, 2-20 ng/ml TNF-*α* were added to the culture medium and incubated for 24 h, respectively. Cultured cells were washed three times with PBS and then 10 scratches were made in a 6-well plate using a sterile pipette tip in the presence of 1 mg/ml Lucifer yellow dye. Next, the cells were incubated in a 37°C incubator for 5 min. The Lucifer yellow was discarded and washed three times with PBS. Subsequently, cells were fixed with 4% PFA for 12 min and observed under a Leica confocal microscopy. GJIC activity was expressed as the number of cells labeled with Lucifer yellow.

### 2.9. Statistical Analysis

The quantitative data was evaluated using an unpaired *t*-test or a one-way analysis of variance ANOVA, and the results are displayed as a mean ± SEM. The statistical significance was assessed by a *p* value less than or equal to 0.05.

## 3. Results

### 3.1. TNF-*α* Disrupts the Structure of Cx43 Mediated Gap Junction in the Rabbit Corneal Endothelium

The impact of TNF-*α* on Cx43 structure in the rabbit corneal endothelium was analyzed by immunostaining. The isolated corneal endothelial tissues were initially treated with 2, 10, or 20 ng/ml TNF-*α* for 24 hours. In the normal control, there was a large gap junction complex mediated by Cx43 in the cornea endothelium (Figure 1(a)). Treatment with a lower concentration of TNF-*α* (2 ng/ml) did not affect the Cx43 mediated gap junction plaques (Figure 1(b)). However, after treatment with a higher concentration of TNF-*α* (10 ng/ml), large gap junction plaques were rarely observed in the corneal endothelium (Figure 1(c)). On the other hand, treatment with 20 ng/ml of TNF-*α* led to the disappearance of typical Cx43 plaques in the endothelial cell border (Figure 1(d)). These results demonstrated that treatment with TNF-*α* induces disruption of Cx43 mediated gap junction of cultured rabbit corneal endothelial tissues in a dose-dependent fashion.

### 3.2. TNF-*α* Attenuates Expression of Cx43 Protein in Rabbit Corneal Endothelium

We employed western blot evaluation to analyze the correlation of the disruption of Cx43 with the differential expression of gap junction proteins. The results showed significant suppression of the expression of Cx43 following exposure to 10 ng/ml (36.8%) and 20 ng/ml TNF-*α* (70%). In contrast, treatment with 2 ng/ml TNF-*α* did not alter the Cx43 expression (Figures 2(a) and 2(b)). These results demonstrated that high concentrations of TNF-*α* reduce the protein expression of Cx43. Since the tight junction marker ZO-1 is pivotal in regulating corneal endothelial barrier properties and gap junction intercellular communication [16, 25], we examined the impact of TNF-*α* on the ZO-1 expression. Western blot findings demonstrated a nonsignificant difference between the normal control group and the TNF- treated group in the amount of ZO-1 protein expression (Figure 2(a)).

### 3.3. Effect of TNF-*α* on Cx43 mRNA Levels in Rabbit Corneal Endothelium

To determine whether Cx43 mRNA expression corresponded with protein expression, the different TNF-*α* treatment concentration groups underwent RT-qPCR analyses. Our findings showed no marked differences in the mRNA expression between the Cx43 and ZO-1 after treatment with lower concentrations of TNF-*α* at 2 ng/ml. Besides, concentrations of TNF-*α* at 20 ng/ml did not also downregulate the expression of Cx43 mRNA (Figures 3(a) and 3(b)). These results suggest that Cx43 may undergo posttranslational modification after exposure to TNF-*α*.

### 3.4. TNF-*α* Reduces the Interaction between ZO-1 and Cx43 in Cultured Rabbit Corneal Endothelium

We previously reported that treatment with TNF-*α* disrupted the tight junction-mediated corneal endothelial barrier function in a dose-dependent manner [24]. The tight junction marker, ZO-1, is crucial in regulating corneal epithelial and endothelial barrier properties. In addition, the interaction within ZO-1 and Cx43 mainly maintains the functions of the gap junction and regulates GJIC activity [4, 24]. Thus, Cx43 and ZO-1 interaction decrease or increase may induce gap junction dysfunction. In order to determine the impact of TNF-*α* on the association between Cx43 and ZO-1, double staining of ZO-1 and Cx43 proteins and immunoprecipitation were used to assess the gap junction integrity. The double immunostaining results showed a marked decline in the binding of ZO-1 with Cx43; large gap junctional complexes were rarely observed in the 10 ng/ml and 20 ng/ml TNF-*α* treated groups (Figures 4(c) and 4(d)). On the other hand, tight binding among ZO-1 and Cx43 was observed in the normal rabbit corneal endothelium (Figure 4(a)). Similarly, a low concentration of TNF-*α* at 2 ng/ml did not destroy the interaction between ZO-1 and Cx43 (Figure 4(b)). Immunoprecipitation results showed that the interaction between ZO-1 and Cx43 was significantly decreased by 29% and 46.1% in the rabbit corneal endothelial cells treated with high concentrations of TNF-*α* compared with the control group (Figures 4(e) and 4(f)). Taken together, these results indicated that TNF-*α* disturbs the connection between ZO-1 and Cx43 in the rabbit corneal endothelium.

### 3.5. TNF-*α* Inhibits GJIC Activity of Primary Rabbit Corneal Endothelial Cells

The SLDT assay is a very important method for evaluating the GJIC activity. To investigate the effect of TNF-*α* on GJIC activity of rabbit corneal endothelial cells, primary cultured rabbit corneal endothelial cells were used in this study. Firstly, cells were treated with different concentrations of TNF-*α* (2-20 ng/ml) for 24 h before the detection of GJIC activity. The SLDT assay was then adopted to determine the number of cells labeled with Lucifer yellow (LY) through gap junctions. The results showed that low concentration of TNF-*α* (2 ng/ml) (Figure 5(b)) did not decrease the activity of GJIC compared with the control group (Figure 5(a)). However, high concentration of TNF-*α* (10, 20 ng/ml) significantly inhibited the activity of GJIC by 47.1% and 64%, respectively (Figures 5(c) and 5(d)). Taken together, we showed that TNF-*α* disrupts GJIC by reducing the association between Cx43 and ZO-1 and downregulating the expression of Cx43.

## 4. Discussion

Human corneal endothelial cells fail to proliferate because of restriction of the cell cycle in G1 phase. A variety of eye diseases such as surgical trauma, cataract surgery, glaucoma, or topically applied of eye preparations could damage corneal endothelial cells, which then induces corneal endothelial dysfunction. Elevated TNF-*α* in various chronic eye diseases contributes a major impact in the dysfunction of corneal endothelial homeostasis. Prior research has demonstrated that TNF-*α* can disrupt the localization and expression of tight junction proteins by phosphorylating myosin light chain kinase (MLCK), leading to corneal endothelial dysfunction in rabbits. We also confirmed that preservative BAK induces gap junction dysfunction by phosphorylating Cx43 and disrupting the association between Cx43 and ZO-1. Although the effect of BAK on the gap junctions has been well demonstrated, the impact of TNF-*α* on the GJIC of corneal endothelium remains unclear.

In this study, we demonstrated that TNF-*α* can damage the Cx43 mediated gap junction structure of the rabbit corneal endothelium and reduce the expression of Cx43 (Figures 1 and 2). Besides, the effect of TNF-*α* on gap junction dysfunction was concentration-dependent (Figure 1). Further analysis showed that the dysfunction of GJIC activity of the rabbit corneal endothelial cells might be due to reduced interaction between the Cx43 and ZO-1 induced by high concentrations of TNF-*α* (Figures 4 and 5).

Although we have demonstrated the role of TNF-*α* in inducing gap junction dysfunction in rabbit corneal endothelium, some mechanisms still need to be explained. For instance, exposure to high concentrations of TNF-*α* downregulated Cx43 protein levels, there have been a nonsignificant variation in the mRNA levels between the different groups (Figure 3). This underlying mechanism is like the previously identified dysfunction of BAK in regulating the gap junctions [9]. We hypothesized that topical application of BAK on the ocular surface might fuel high expression of TNF-*α* in aqueous humor, thus accelerating the disruption of the function of the corneal endothelial gap junction. These common results suggest that posttranslational activities of Cx43 may modulate disruption of the gap junctions by TNF-*α*. Therfore, we speculated that this may be a common feature of TNF-*α*-related signaling induced corneal endothelial gap junction dysfunction. Consequently, the downregulation of Cx43 and the disruption of the tight junction marker, ZO-1, contribute to the TNF-*α*-caused malfunction of GJIC in the corneal endothelium.

TNF-*α* plays a bidirectional role in regulating GJIC mediated by Cx43. Lin et al. revealed that TNF-*α* could upregulate the expression of Cx43 and promote the proliferation of aortic smooth muscle cells [26]. In addition, Lagos-Cabre et al. demonstrated increased Cx43 expression in astrocytes after TNF-*α* treatment [27]. On the other hand, Kabatkova et al. showed that TNF-*α*-treated rat hepatocytes caused downregulation of the Cx43 expression and inhibited GJIC of hepatocytes [28]. Our study revealed that TNF-*α* treatment reduces Cx43-mediated GJIC in rabbit corneal endothelium. Therefore, the effect of TNF-*α* on gap junction function may be different in different tissues or cells and thus needs further research to identify the underlying specific mechanism.

The regulation of gap junctions is significantly impacted by the cooperation between ZO-1 and Cx43. To exert its biological effect, the C-terminal of the Cx43 protein binds the PDZ2 structure of ZO-1 [29–31]. Previous studies reported that Cx43 interacts with ZO-1 to regulate cell migration in cerebral endothelial wound healing [30]. The structure and stability of the gap junction channel can be controlled by a complex that consists of Cx43 and ZO-1 [32]. In this study, we demonstrated that TNF-*α* inhibits rabbit corneal endothelial GJIC by decreasing the interaction between ZO-1 and Cx43, downregulating the expression of Cx43 and disrupting the distribution of Cx43. However, this research still has some limatations. For example, how TNF-*α* downregulates the interaction between ZO-1 and Cx43 remains undertemined, a more detailed mechanism still needs to be elaborated in the future. In fact, we have detected TNF-*α*-related classical NF-*κ*B, JNK, and AKT signaling pathways in previous experiments. Unfortunately, no significant activation of the related signaling pathways was detected. Due to the special anatomy of the cornea, the corneal endothelium is directly exposed to aqueous humor. However, Cx43-mediated gap junction and the barrier integrity of the endothelium are effective in maintenance of stromal deturgescence and corneal transparency. When patients with endophthalmitis, uveitis, and other ocular trauma, the level of TNF-*α* will rise sharply in aqueous humor. Due to the direct physical contact between aqueous humor and corneal endothelium, we hypothesized that high concentrations of TNF-*α* may act directly on Cx43 protein, disrupt the interaction between ZO-1 and Cx43, and downregulate the expression level of Cx43 to disrupt corneal endothelial gap junctional intercellular communication (GJIC). We are well aware of the limitations of this study and will continue to explore the specific mechanisms and potential drugs that protect GJIC of corneal endothelial cells in the future.

## 5. Conclusions

In conclusion, we examined the impact of TNF-*α* on the corneal endothelial gap junction. Our findings demonstrated that TNF-*α* could disrupt the gap junctional intercellular communication (GJIC) of rabbit corneal endothelium by disturbing the connection between Cx43 and ZO-1, downregulating the expression of Cx43, and destroying the distribution of Cx43. The gap junction plays a crucial part in regulating corneal endothelial cell homeostasis. Additionally, the current investigation elucidates the effect of stimulation of TNF-*α* on Cx43-mediated GJIC in the corneal endothelium. It offers a new basis for the therapy of the corneal endothelial malfunction induced by elevated TNF-*α* in various eye diseases.

## Figures and Tables

**Figure 1:** Impact of TNF-*α* on Cx43 distribution in rabbit corneal endothelium. (a) Cx43 distribution in normal rabbit corneal endothelium. (b) Cx43 distribution in rabbit corneal endothelium treated with 2 ng/ml TNF-*α*. (c) Cx43 distribution in 10 ng/ml TNF-*α* treated rabbit corneal endothelium. (d) Cx43 distribution in 20 ng/ml TNF-*α* treated rabbit corneal endothelium. DAPI: blue color; Cx43: red color; and scale bar: a − d = 5 *μ*m (*n* = 6 rabbits per group).

**Figure 2:** Impact of TNF-*α* on Cx43 and ZO-1 protein expression in rabbit corneal endothelium. (a) The expression of Cx43 and ZO-1 protein in different concentrations of TNF-*α*-treated rabbit corneal endothelium. (b) Quantification of the Cx43 protein expression in different TNF-*α* treatment groups. (*n* = 6 rabbits per group; mean ± SEM, ∗∗ represented *p* < 0.01 vs. control, and ∗∗∗ represented *p* < 0.001 vs. control).

**Figure 3:** Impact of TNF-*α* on Cx43 and ZO-1 mRNA expression in rabbit corneal endothelium. (a) Quantifying Cx43 mRNA expression in normal rabbit corneal endothelium and TNF-*α* treatment groups. (b) Quantifying ZO-1 mRNA expression in normal rabbit corneal endothelium and TNF-*α* treatment groups. (*n* = 6 rabbits per group; mean ± SEM).

**Figure 4:** Reduced association between Cx43 and ZO-1 in the TNF-*α*-treated corneal endothelium. (a) Cx43 (red color) and ZO-1 (green color) double staining in normal rabbit corneal endothelium. (b) Cx43 (red color) and ZO-1 (green color) colocalization in 2 ng/ml TNF-*α*-treated rabbit corneal endothelium. (c) Cx43 (red color) and ZO-1 (green color) colocalization in 10 ng/ml TNF-*α*-treated rabbit corneal endothelium. (d) Cx43 (red color) and ZO-1 (green color) interaction in 20 ng/ml TNF-*α*-treated rabbit corneal endothelium. Scale bar: a − d = 5 *μ*m (*n* = 6 rabbits per group). (e) Immunoprecipitation indicated changes in the interaction of Cx43 with ZO-1 in different TNF-*α* treatment groups. (f) Quantification of the ratio of ZO-1 to Cx43 in different TNF-*α* treatment groups. (*n* = 6 rabbits per group; mean ± SEM, ∗∗ represented *p* < 0.01 vs. control, and ∗∗∗ represented *p* < 0.001 vs. control).

**Figure 5:** TNF-*α* treatment inhibited GJIC activity of primary cultured rabbit corneal endothelial cells. (a) LY-labeled cells in normal rabbit corneal endothelial cells. (b) LY-labeled cells in 2 ng/ml TNF-*α*-treated normal rabbit corneal endothelial cells. (c) LY-labeled cells in 10 ng/ml TNF-*α*-treated rabbit corneal endothelial cells. (d) LY-labeled cells in 20 ng/ml TNF-*α*-treated rabbit corneal endothelial cells. (e) Quantifying GJIC activity in normal rabbit corneal endothelial cells and TNF-*α* treatment groups. (*n* = 6 rabbits per group; mean ± SEM, scale bar = 10 *μ*m, ∗∗∗ represented *p* < 0.001 vs. control, and ∗∗∗∗ represented *p* < 0.0001 vs. control).

## Data Availability

All experimental data supporting this study are available from the corresponding author upon reasonable request.
